# The Infection Control Route in the Operating Room Effectively Reduces the Wound Infection of Patients

This article has been retracted.

**DOI:** 10.1155/2022/9270045

**Published:** 2022-06-06

**Authors:** Xiufang Tang, Zhenqing Ren, Yueqin Miao, Hongmei Dou

**Affiliations:** ^1^Department of Operating Room, Taizhou People's Hospital, Taizhou, Jiangsu, China; ^2^Nursing Department, Taizhou People's Hospital, Taizhou, Jiangsu, China

## Abstract

Surgical care is one of the significant aspects of global healthcare, with approximately 234 million operations being conducted annually. Surgical treatment has a substantial risk of complications and death. This study was conducted to explore the application effect of the infection control route in the operating room on the wound infection prevention care of patients. The clinical data of 136 patients receiving surgical treatment from October 2018 to October 2019 were retrospectively analyzed. The participants were assigned via random draw at a ratio of 1 : 1 to receive either routine care management (control group) or the infection control route (research group). The surgical wound infections of patients in the two groups were compared. The research group had higher scores in surgical materials management and disinfectant management than the control group (*P* < 0.01). In the research group, the total number of colonies within 5 minutes before surgery, 25 minutes after the start of surgery, and after surgery were all smaller than those in the control group (*P* < 0.01). There were no significant differences in the grade B healing rate between the two groups (*P* > 0.05), and the research group had a significantly higher healing rate in grade A than the control group, but its grade C healing rate and wound infection rate were significantly lower than those in the control group (*P* < 0.05). In the research group, the length of hospital stay, the time to get out of bed, the antibiotic use duration, and the stitch removal time was significantly shorter than those in the control group (*P* < 0.0001). The research group received a higher clinical nursing satisfaction than the control group (*P* < 0.05). The infection control route in the operating room for infection prevention care effectively reduces the wound infection rate of patients and accelerates their postoperative recovery.

## 1. Introduction

Surgical care is one of the significant aspects of global healthcare, with approximately 234 million operations being conducted annually. Surgical therapy has a substantial risk of complications and death. Research has reported that one out of every 150 inpatients' death is attributed to adverse events among which surgical therapy accounts for nearly two-thirds of in-hospital incidents [1]. Surgical wound infection, a common surgical complication, is divided into wound infection, deep organ infection, and fascial space infection according to different infection sites. It is caused by exogenous surgical site infection and endogenous surgical site infection [2, 3]. Wound infection compromises the treatment efficacy of patients and causes medical disputes and conflicts.

The operating room is a place with a high risk of disease infection and virus transmission. In the operating room, patients are susceptible to a variety of factors that may lead to wound bleeding and septicemia, so infection control in the operating room is an important measure to effectively prevent and reduce wound infections in patients [4–6].

Currently, invasive treatment is the main surgical measurement. Incomplete disinfection of the operating room, nonstrict implementation of aseptic operations, and an increase in the number of resistant viruses in the air will increase the incidence of wound infection. Efficient modern medical management concepts have fostered an infection control route in the operating room, providing effective preventive measures in improving surgical treatment outcomes and reducing wound infections. The infection control route provides thorough cleaning and disinfection of the operating room, and improves the surgical infection control concepts and skills of the medical staff, offering better surgical care services [7, 8].

Accordingly, this study was undertaken to explore the effect of the infection control route in the operating room on the wound infection prevention care of patients. The operating room infection control approaches are used for wound infection prevention care, which may significantly reduce wound infection, speed up postoperative recovery, and increase nurse satisfaction. The experimental outcomes and significance of this study exceeded those of the earlier approaches.

The remaining organization of the paper is as follows: Section 2 describes the materials and methods used in this research.  Section 3 shows the result of the study in different groups. A comprehensive discussion is presented in Section 4.  Section 5 summarizes the overall theme of the paper.

## 2. Materials and Methods

### 2.1. General Materials

The clinical data of 136 patients receiving surgical treatment from October 2018 to October 2019 were retrospectively analyzed. The participants were assigned via random draw at a ratio of 1 : 1 to receive either routine care management (control group) or the infection control route (research group). This study was approved by the Ethics Committee of Taizhou People's Hospital, no.TZH397.

### 2.2. Inclusion Criteria

Patients without surgical contraindications, aged ≥18 years, and who provided written informed consent were included.

### 2.3. Exclusion Criteria

Patients with severe brain, heart, kidney, and other organ diseases or abnormal immune and hematopoietic functions; with the withdrawal of consent; who died; who failed to cooperate with the study; with communication or mental and cognitive disorders; with infectious diseases were excluded.

### 2.4. Methods

The control group received routine care management in the operating room. On the day before surgery, patients and their families were given surgical precautions, and the patients were prohibited from food and drinks. The research group received the infection route in the operating room.

1. The patient's condition was thoroughly evaluated and detailed information was collected before the operation. A targeted program was developed for malnourished patients to improve their immunity for full preparation for postoperative prevention of wound infection.
2. One day before the operation, the patients were informed of the purpose, procedure, and precautions of the surgery, and a comprehensive physical examination was conducted. Patients who were nervous and anxious before the operation were actively communicated to eliminate negative emotions and help them establish a positive mental state.
3. The self-cleaning system was turned on 30 minutes before surgery to maintain the operating room temperature at 21–25°C and relative humidity at 30–60%.
4. The skin of the surgical area was strictly disinfected before surgery, and the wound was covered with a protective film. After incision, a protector was used to prevent internal infection with strict aseptic practice. The wound was rinsed successively with iodophor and saline during suturing, and hypothermia in the perioperative period was prevented. (5) During surgery, the circulating nurse specifically directed and supervised the surgical care, especially the management of sterile items and aseptic operation. If the surgeon's gloves were damaged or punctured by instruments, the gloves should be replaced immediately. The self-cleaning time between two surgeries was ensured to meet the requirements. (6) Professional skills training was conducted monthly for the medical staff in the operating room, and monthly tests on the prevention and treatment of wound incision infections were organized to improve the professional skills of the medical staff.

Infection control path:

1. Layout and process control: According to the actual situation of the hospital, the surgical channel, staff channel, and article channel were strictly distinguished, and signs were given at prominent locations to fully avoid potential infection factors.
2. Physician infection control: during surgery, personnel must be restricted to enter and exit the operating room according to requirements, with visitors limited to two people, with special caps in strips instead of ordinary and floral cotton caps. Strict intraoperative asepsis was required. A “no entry” sign was placed at the entrance of the operating room to reduce the rate of surgical infection.
3. Infection control of the operating room environment and apparatus: items in the operating room should be as streamlined as possible and kept clean. Special personnel were arranged to clean the items and floors of the operating room after surgery. Surgical instruments and items used by doctors must be strictly sterilized and disinfected before they were brought into the operating room. Dedicated personnel were arranged to clean the items and floors of the operating room after surgery.

Prevention of incisional infections in patients using traditional Chinese medicine (TCM) nursing.

1. TCM evidence-based care: according to the changes of the four seasons, the daily care of patients was adjusted to follow the four seasons and balance yin and yang. In spring, the patients are encouraged to maintain a relaxed mood, follow a diet with more sweet foods, less sour foods, and avoid oily and spicy foods, and have a healthy lifestyle. In summer, patients are advised to maintain a calm state of mind, and to eat foods that clear the heart and fire and relieve the heat, and to avoid cold, unclean, fatty, and spicy foods. They are also advised to sleep early and get up early. In autumn, patients are advised to avoid sadness and grief, and to follow a diet based on moistening the lungs and generating fluids, with vegetables and fruits, and avoiding spicy and hot foods. They were advised to sleep early and get up late. In winter, patients should avoid panic, and the diet should contain warm foods and avoid cold and salty foods. Back tapping care can also be introduced to the patients: The patient was tapped along the spine and bilateral Zutaiyang bladder meridians along the spine from top to bottom for 20 min, with slow movements to avoid choking and coughing. It was performed twice daily.
2. Acupressure on the Tiandu acupoint: the patient was kept in a recumbent or sitting position, and the massage therapist held the patient's back with one hand and placed the other hand on the patient's Tiandu point in the superior sternal fossa and pressed the Tiandu point with the index finger and middle finger to induce the patient to cough; this promotes sputum excretion. The acupressure was performed twice daily for 2–5 min each time. The treatment should be discontinued in the event of an irritating cough.

### 2.5. Evaluation Indexes

The clinical data of patients in the two groups such as gender, age, weight, type of surgery, and education level were compared. The *Operating Room Management Score Scale* [9] was employed to evaluate the operating room management of the two groups, and the scale included the materials management score and disinfection management score, with 100 points for each item. The higher the score, the higher the quality of operating room management.

Colony samples 5 min before the operation, 25 min after the start of the operation, and after the operation were detected. Agar medium (Ф90 mm) sampling points were set up in the operating area and surrounding area of the operating room, with the sampling point at 0.8 m above the ground. The medium was sent for inspection after 30 min of sampling and was cultivated in a greenhouse at 36–38°C for 48 hours, followed by observation of the culture results. The total number of colonies = 50000 average number of colonies/medium area × medium exposure time [10].

The following grades were used to classify the healing conditions of the surgical wound: Grade A: the postoperative wound was healed well without exudation, effusion, and hematoma. Grade B: the wound was basically healed, with slight exudation, effusion, and hematoma but no suppuration. Grade C: the wound was in a poor state, with exudation, effusion, hematoma, and suppuration. The wound infection rate of the two groups was counted.

The length of hospital stay, operation time, antibiotic use time, and stitch removal time of patients in the two groups were recorded and compared. The *Clinical Nursing Satisfaction Questionnaire for Surgical Patients* made by our hospital was used to evaluate the clinical care status of the two groups, and the results of the questionnaire are divided into highly satisfied, satisfied, and dissatisfied.

### 2.6. Statistical Methods

SPSS21.0 software was used for data analysis. The enumeration data are expressed as (n (%)) and analyzed using the chi-square test, and the measurement data are expressed as mean ± SD and analyzed using the *t*-test. Differences were considered statistically significant at *P* < 0.05.

## 3. Results

This section represents the experimental results attained in the conduction of this study. The result of the study is evaluated in different groups to clarify the impact of these factors on the results.

### 3.1. Comparison of Clinical Data

There were no significant differences in the baseline characteristics between the two groups (*P* > 0.05) (Table 1).

### 3.2. Comparison of Nursing Quality Scores

The research group had significantly better scores on item management and disinfection management as compared to the control group (*P* < 0.05) (Figure 1).

### 3.3. Comparison of Colony Numbers at Different Time Points

In the research group, the total number of colonies within 5 minutes before surgery, 25 minutes after the start of surgery, and after surgery were all smaller than those in the control group (*P* < 0.05) (Table 2).

### 3.4. Comparison of Healing and Infection of Wounds

There were no significant differences in the grade B healing rate between the two groups (*P* > 0.05), and the research group had a significantly higher healing rate in grade A than the control group, but its grade C healing rate and wound infection rate were significantly lower than those of the control group (*P* < 0.05) (Table 3 and Figure 2).

### 3.5. Comparison of Postoperative Conditions

In the research group, the length of hospital stay, the time to get out of bed, the antibiotic use duration, and the stitch removal time was significantly shorter than those of the control group (*P* < 0.0001) (Table 4).

### 3.6. Comparison of Clinical Nursing Satisfaction

The research group received a higher clinical nursing satisfaction than the control group (*P* < 0.05) (Table 5 and Figures 3 and 4).

## 4. Discussion

Effective prevention of surgical wound infection is critical to patient safety and postoperative recovery [11]. With the continuous development of medical technology, the facilities in the operating room have been significantly upgraded, and stricter requirements for the management of the operating room have also been proposed. Efficient operating room management ensures the smooth implementation of the operation and reduces wound infection. In recent years, there has been a significant increase in reports about surgical infections, which results in increased psychological pressure on patients and their families [12,13]. The decreased immune function of patients during surgery, coupled with the invasive nature of surgery, predisposes them to infections, which may result in aggravated disease conditions, increased the workload of medical staff, and more consumption of medical resources. Therefore, effective infection control routes in the operating room contribute substantially to improving the treatment efficacy, relieving patients' pain, and reducing medical resources waste [14–16].

It has been reported that [17] the total colonies numbers in the air in the general surgical operating room should be ≤200 cfu/m3. A significant number of clinical examinations had shown that inadequate air quality in the operating room is mainly attributed to poor air circulation due to poor handling of medical equipment and sterilized items in the operating room, absence of strict sterilization of medical equipment before use, and violation of the rules of aseptic operation [18, 19].

Accordingly, a targeted infection control route in the operating room was formulated in the present study, to prevent the wound infection and improve the treatment efficacy.

The results of the present study revealed that the wound infection rate of patients treated with the infection control route in the operating room was 2.94%, which was significantly lower than 13.24% in the control group. The wound healing efficacy of the observation group was also higher than that of the control group. The wound healing grade refers to the evaluation of the healing degree according to conditions during healing, which objectively reflects the postoperative rehabilitation efficacy [20]. Fitriani et al. [21] demonstrated that the infection control management in the operating room was applied to the groin wound infection, and the overall infection rate (including superficial wound infection) was 3.03%, which was lower than 14.22% in the control group, indicating that the infection control route in the operating room significantly reduced wound infection and improved the treatment efficacy. Furthermore, the infection control route effectively reduced the wound infection rate, accelerated postoperative recovery, and improved nursing satisfaction. TCM nursing is the application of TCM discriminative ideas and meridian medicine for care [9]. TCM believes that in order to prolong life and maintain health, human beings should be in harmony with nature, eat and drink in a disciplined manner, and live in a regular manner. Therefore, it is a special part of TCM care to adapt the patient's living conditions to nature. Regularity in rising and living includes conformity to the four seasons, nurturing Yang in spring and summer, nurturing Yin in autumn and winter, as well as avoiding deficient evil and thieving wind at times, thereby harmonizing the body's yin and yang, promoting the body's recovery, improving the body's immune system, and avoiding the invasion of evil spirits [10]. In addition, the patient's mood changes are one of the key elements of TCM care. According to TCM, the seven emotions enter the five viscera, and any excess of the seven emotions will lead to diseases of the internal organs. Therefore, it is necessary to appropriately manage the patient's emotions and maintain a calm state of mind, which is conducive to the recovery of the patient. The increased resistance of patients to diseases facilitates the recovery from a hypertensive cerebral hemorrhage and also prevents complications [11].

## 5. Conclusion

The infection control route in the operating room for infection prevention care effectively reduces the wound infection rate of patients and accelerates their postoperative recovery.

## Figures and Tables

**Figure 1:** Comparison of nursing quality (*x* ± *s*). *Note.* In Figure 1, the *x*-axis represents the item management score and disinfection management score, and the *y*-axis shows the score and points. The item management score and disinfection management score in the research group were 96.74 ± 2.03 points and 98.03 ± 1.25 points, respectively. The item management score and disinfection management score in the control group were 91.36 ± 2.16 points and 92.76 ± 1.36 points, respectively. There is a significant difference in the item management score between the two groups (*t* = 14.967, ^*∗*^*P* < 0.05). There is a significant difference in the disinfection management scores between the two groups (*t* = 23.526, ^*∗*^*P* < 0.05).

**Figure 2:** Comparison of healing and infection of the incision.

**Figure 3:** Overall nurse satisfaction.

**Figure 4:** Total satisfaction.

**Table 1:** Comparison of clinical data.

Factors	Research group (*n* = 68)	Control group (*n* = 68)	*X* ^2^/*t*	*p*
Gender				
Male	36	35	0.030	0.864
Female	32	33		
Average age (years, *x* ± *s*)	43.75 ± 3.42	43.48 ± 3.35	0.465	0.643
Average weight (kg, *x* ± *s*)	67.34 ± 5.63	67.42 ± 5.49	0.084	0.933
Type of surgery				
Orthopedics	13	15	0.180	0.671
Intestines and stomach	8	10	0.634	0.426
Urology	16	19	0.346	0.556
Liver and gallbladder	17	14	0.376	0.540
Gynecology	14	10	0.810	0.368
Incision classification				
I	13	14	0.046	0.830
I	38	40	0.120	0.729
III	17	14	0.376	0.540
Education				
Specialist education or above	18	21	0.324	0.569
High school	35	37	0.118	0.731
Middle school or below	15	10	1.225	0.268

**Table 2:** Comparison of colonies numbers at different time points (cfu/30 minФ90,*x* ± *s*).

Group	n	5 min before operation		30 min after the start of operation		After operation	
		Surgery area	Adjacent area	Surgery area	Adjacent area	Surgery area	Adjacent area
Research group	68	0.82 ± 0.63	1.98 ± 1.02	3.87 ± 1.17	5.13 ± 2.03	6.96 ± 3.28	8.77 ± 4.06
Control group	68	2.05 ± 0.78	3.53 ± 1.21	5.01 ± 1.36	6.32 ± 2.37	8.24 ± 3.97	10.33 ± 4.19
t		10.116	8.077	5.241	3.145	2.05	2.205
p		0.001	0.002	0.002	0.002	0.042	0.029

**Table 3:** Comparison of healing and infection of the incision (n (%))

Group	n	Grade A healing	Grade B healing	Grade C healing	Incision infection rate
Research group	68	**63 (92.65)**	**4 (5.88)**	**2 (2.94)**	**2 (2.94)**
Control group	68	**58 (85.29)**	**8 (11.77)**	**12 (17.65)**	**9 (13.24)**
*X* ^*2*^		1.873	1.462	7.963	4.847
p		0.171	0.227	0.005	0.028

**Table 4:** Comparison of the postoperative conditions (d, *x* ± *s*).

Group	n	Hospitalization time	The time to get out of bed at first	The time of antibiotic use	The time of stitch removal
Research group	68	8.32 ± 2.18	2.53 ± 0.75	2.33 ± 0.65	6.72 ± 1.47
Control group	68	11.16 ± 1.03	3.72 ± 0.83	4.53 ± 0.87	8.93 ± 1.54
t		9.713	8.772	16.705	8.560
p		**<0.0001**	**<0.0001**	**<0.0001**	**<0.0001**

**Table 5:** Comparison of clinical nursing satisfaction (n (%)).

Group	n	Highly satisfied	Satisfied	Dissatisfied	Total satisfaction
Research group	68	49 (72.06)	18 (26.47)	1 (1.47)	67 (98.53)
Control group	68	42 (61.76)	19 (27.94)	7 (10.29)	63 (92.65)
*X* ^2^					4.781
p					0.029

## Data Availability

The findings of this study are available from the corresponding author upon request.
